The article "Psychotherapy Combined with Western Medicine in the Treatment of Children with Tic Disorder: Systematic Review and Meta-Analysis" was retracted in 2023. Reasons: suspected computer-generated content; unreliable results or conclusions; concerns about the data; concerns about the results or conclusions.

# Psychotherapy Combined with Western Medicine in the Treatment of Children with Tic Disorder: Systematic Review and Meta-Analysis

**DOI:** 10.1155/2022/2365210

**Published:** 2022-04-04

**Authors:** Yamin Kong, Xueyuan Zhang, Bingxiang Ma

**Affiliations:** The First Affiliated Hospital of Henan University of Traditional Chinese Medicine, Zhengzhou, 450000 Henan, China

## Abstract

**Objective:**

To evaluate the efficacy of psychotherapy in children with tic disorder and to provide basis for the application of psychotherapy in the treatment of children with tic disorder.

**Methods:**

A detailed search was conducted based on PubMed, Cochrane library database, CNKI, Wanfang Data, and VIP database to determine the randomized controlled trial (RCT) of psychotherapy combined with drugs and oral drugs in the treatment of tic disorder. The search time was from the establishment of the database to August 20, 2021. All kinds of extracted data are meta analyzed, and the statistical software used is Review Manager 5.3 software.

**Results:**

According to the inclusion and exclusion criteria, 14 clinical trials were finally included, including 513 TD children, including 267 in the psychological intervention group and 246 in the control group. All trials were conducted in China and published from 2013 to 2021. In terms of clinical efficacy, compared with the control group, the psychotherapy combined with drugs group had more advantages in improving the effective rate (RR = 3.25, 95% CI: 2.17~4.85, *Z* = 5.74, *P* < 0.00001) and improving the clinical symptoms of children with TD (WM = −5.36, 95% CI: -6.41 ~ -4.30, *Z* = 9.97, *P* < 0.00000 1).

**Conclusion:**

Psychotherapy as an adjuvant therapy for clinical treatment of TD can improve the clinical efficacy, but due to the low methodological quality of the existing trials, the research may have potential bias. In the future, large sample, multicenter, and double-blind randomized controlled trials need to be carried out to provide further support.

## 1. Introduction

Tic disorders (TD) are a common neurodevelopmental disorder in childhood. The onset age of the disease is mostly between 3 and 14 years old, and the prevalence rate of boys is 2-4 times higher than that of girls. It is mainly manifested in involuntary, repeated, and rapid muscle movement twitch and vocal twitch in one or more parts [1], such as frequent blinking, eyebrow squeezing, nose sucking, mouth nubbing, and strange cry. In recent years, the incidence rate is increasing year by year. The etiology and pathogenesis of the disease are not fully understood. Most studies believe that the incidence of tic disorder is related to heredity, neurotransmitter balance, neurodevelopmental defects, abnormal brain structure or function, infection immunity, and mental and psychological environment. At present, there is no perfect treatment plan for tic disorder at home and abroad. The clinical treatment methods mainly focus on drugs, such as haloperidol, aripiprazole, risperidone, tiapride hydrochloride, and clonidine. Although the clinical symptoms can be temporarily controlled, there are many extrapyramidal reactions and other side effects, and it is easy to relapse after drug withdrawal [2–4].

In recent years, some scholars have suggested using comprehensive treatment methods to treat children with tic disorder, including acupuncture, traditional Chinese medicine, and psychological intervention [5–7]. Among them, psychotherapy belonging to nondrug therapy highlights its unique advantages, but it has not been widely used in the international medical system. Psychotherapy mainly includes cognition, behavior, and family intervention [8]. Studies have found that tic symptoms can be aggravated by adverse emotional factors such as anxiety, anxiety, excitement, and impulse and relieved by emotional relief [9]. The use of psychotherapy can alleviate emotions and achieve the purpose of treatment [10]. In order to explore whether psychological intervention combined with drug therapy has curative effect advantages compared with western medicine alone, this study collected and sorted out the randomized controlled trials of psychological intervention in the treatment of tic disorder published at home and abroad for quality evaluation and meta-analysis and refined the high-quality evidence, in order to provide evidence-based basis for the curative effect advantages of psychological intervention in the treatment of tic disorder and provide guidance for clinical diagnosis and treatment.

## 2. Materials and Methods

### 2.1. Inclusion Criteria

#### 2.1.1. Research Design

RCT of psychotherapy is combined with drug therapy in children with TD.

#### 2.1.2. Research Object

Both the experimental group and the control group were children (age < 18 years), regardless of gender and race. The diagnostic criteria may be from the Diagnostic and Statistical Manual, the Third Edition (DSM-III), the Fourth Edition (DSM-IV), or the revised version of the Fifth Edition (DSM-V); International Classification of Diseases 10th Edition (ICD-10), 11th Edition (ICD-11); Chinese Classification of Mental Disorders Second Edition (CCMD-2) and Third Edition (CCMD-3); or other clearly defined diagnostic criteria. There was no significant heterogeneity in general data and baseline characteristics between the two groups.

#### 2.1.3. Intervention Measures

The control group was treated with drugs, including haloperidol, aripiprazole, risperidone, tiapride hydrochloride, and clonidine, on the basis of the control group, the experimental group adopted psychotherapy intervention, including supportive psychotherapy, family psychological intervention, cognitive therapy, behavior intervention, and exposure and response prevention.

#### 2.1.4. Outcome Indicators

At least include the total effective rate of psychotherapy combined with drugs in the treatment of TD, Yale Global Tie Severity Scale (YGTSS), and the outcome criteria are recognized and clear.

### 2.2. Exclusion Criteria

(1) Review, experience summary, theory, discussion, case report, experimental research, and other types of literature; (2) the trial design did not conform to the randomized control principle specified in this study; (3) the subjects did not meet the diagnostic criteria of TD or were complicated with attention deficit hyperactivity disorder, autism, epilepsy, and other diseases; (4) For different literatures and repeated published studies published in the same study, the first published one is selected, and the English literature of Chinese-English bilingual literature is excluded.

### 2.3. Result Evaluation Type

#### 2.3.1. Main Indicators

YGTSS score. YGTSS included 30 items, including 18 categories of motor and vocal twitch, self-mutilation behavior, anger control problems, and a severity rating scale.

#### 2.3.2. Secondary Indicators

Efficient. Studies that divide the efficiency results into dichotomous methods (effective or ineffective) are taken into account. In some studies, patients with a YGTSS reduction rate of less than 30% were considered “ineffective” and others were considered “effective.” These studies are included in this paper.

### 2.4. Retrieval Strategy

Search PubMed, EMBASE, Web of Science, Cochrane Library, Chinese biomedical literature database (CBM), CNKI, Wanfang Database, and VIP. The retrieval time limit is from database establishment to August 20, 2021.

Using the combination of subject word retrieval, partial free word retrieval, and truncated word retrieval, the Chinese retrieval keywords are tic syndrome, children's tic syndrome, Tourette's syndrome, tic, psychotherapy, behavior therapy, cognition, family, and psychology. English search keywords: tic disorder, transient tic disorders, Tourette syndrome, Tourette disease, Tourette's disease, Tourette, tic, psychotherapy, psychological therapy, cognitive therapy, acceptance and commitment therapy, etc. Subject and free word retrieval are carried out according to different database characteristics. Take PubMed database as an example: #1 = (Tic Disorders OR Transient Tic Disorders OR Tourette Syndrome OR Tourettes Disease OR Tourette's Disorder OR Tourette ORTic), #2 = (Psychotherapy OR Psychological therapy OR Cognitive Therapy OR Acceptance OR Commitment Therapy), #3 = clinical trial, #4 = #1AND#2AND#3. In addition, the references and related reviews included in the study were traced to supplement the relevant literature.

### 2.5. Literature Screening and Data Extraction

Literature screening and data extraction were completed by two researchers independently. The literature screening is determined by two researchers after independent screening according to the inclusion and exclusion criteria of the literature. If there are differences in the inclusion of the literature, the third party will decide whether to include it. Then, the literature data are extracted. The content of literature data extraction mainly includes title, author's name, publication year, random method, sample size of study group and control group, intervention method, and outcome evaluation index.

### 2.6. Literature Quality Evaluation

According to Jadad scoring standard [11], all included literatures were scored in three aspects: (1) randomization of the research scheme (2 points): 2 points for those who generate random numbers by using random number table or computer, 1 point for those who mention two groups of random grouping but do not mention specific random methods, and 0 point for nonrandom experimental design; (2) for the application of the principle of double-blind method (2 points): 2 points will be given if the specific method of blind method is described, 1 point will be given if only the blind method is recorded but not detailed, and 0 point will be given if the blind method is not mentioned or the method is inappropriate; (3) record the abscission of the research object (1 point): 1 point for recording the number of cases related to withdrawal and loss of follow-up, and 0 point for not mentioning withdrawal and loss of follow-up. Those with Jadad score less than 3 are classified as low-quality literature, and those with Jadad score ≥ 3 are classified as high-quality literature (Table 1).

## 3. Statistical Analysis

The extracted data were meta-analyzed with Review Manager 5.3 software recommended by Cochrane. Heterogeneity test: Using *χ*^2^ test and *I*^2^ value to analyze the heterogeneity. If *P* > 0.1 and *I*^2^ ≤ 50%, there is no statistical heterogeneity between the studies. Select the fixed-effect model for meta-analysis; If *P* ≤ 0.1 and *I*^2^ > 50%, it means that there is great statistical heterogeneity between studies. The random effect model is selected for meta-analysis. Counting data: relative risk (RR) and its 95% confidence interval (CI) are used as effect scale indicators. Measurement data: weighted mean (WM) and its 95% confidence interval (CI) are used. Bias analysis: draw a funnel chart. If the funnel chart is asymmetric, it indicates that there is an offset in the data. The more obvious the asymmetry is, the greater the offset degree is.

## 4. Technology Roadmap

A total of 221 literatures were obtained, including 127 in English and 94 in Chinese; finally, 14 papers were included, all of which were conducted in China. The document screening process is shown in Figure 1. A total of 513 TD children were included in 14 literatures, including 267 in the psychological intervention group and 246 in the control group. The basic characteristics of the included literature include (1) general research information, (2) sample size and gender ratio, (3) age, (4) interventions, see Table 2.

## 5. Evaluation of Meta-Analysis Results

### 5.1. Meta-Analysis of Total Effective Rate

Of the 14 literatures, 8 reported the total effective rate [12, 14, 15, 18, 20, 23–25], including 870 patients (433 in the observation group and 437 in the control group). There was homogeneity among the studies (*χ*^2^ = 2.54, *P* = 0.92, *I*^2^ = 0%). The fixed-effect model was used for meta-analysis, and the difference was statistically significant (RR = 3.25, 95% CI: 2.17~4.85, *Z* = 5.74, *P* < 0.00001), see Figure 2.

### 5.2. Meta-Analysis of YGTSS Score after Treatment

Among the 14 literatures, 11 reported the YGTSS score after treatment [5–16], including 1094 patients (544 in the observation group and 550 in the control group). There was heterogeneity among the studies (*χ*^2^ = 28.55, *P* = 0.001, *I*^2^ = 65%). The YGTSS score of the study group was significantly lower than that of the control group after treatment, and the difference was statistically significant (WM = −5.36, 95% CI: -6.41~ -4.30, *Z* = 9.97, *P* < 0.00000 1), see Figure 3.

### 5.3. Publication Bias

In stata14 software, the funnel diagram of efficiency index indicates that it is basically symmetrical, see Figure 4 below.

## 6. Discuss

The results of this study involved 14 randomized controlled trials and 513 patients. The researchers evaluated the quality of the included literature and the risk of bias. The following conclusions can be drawn: compared with the control group (treated with conventional Western Medicine), TD patients randomly assigned to the psychological intervention group showed higher clinical efficacy (RR = 3.25, 95% CI: 2.17~4.85, *Z* = 5.74, *P* < 0.00001) and reduced the total score of YGTSS (WM = −5.36, 95% CI: -6.41 ~ -4.30, *Z* = 9.97, *P* < 0.00000 1). It shows that psychological intervention can improve the clinical symptoms of TS patients and can be used as an adjuvant therapy for TD in clinical practice.

However, this study also has some shortcomings: (1) according to Jadad score, the included literatures are all low-quality literatures, lacking the support of large samples and multicenter high-quality literatures. (2) There are different degrees of methodological problems in the included literature. For example, due to the particularity, diversity, and complexity of psychological intervention treatment, it is difficult to carry out double-blind research, resulting in the low level of relevant research and relevant clinical evidence. (3) There is no description of allocation concealment in the included literature, and there is no explanation for the loss of follow-up and withdrawal cases. It is unclear whether there are other biases, and there is no mention of adverse reactions, which may exaggerate the efficacy of psychotherapy. (4) In the included literature, the inclusion criteria, exclusion criteria, diagnostic criteria, efficacy criteria, and treatment schemes are different, and the data are lack of consistency. (5) The long-term efficacy of psychotherapy was not discussed in the included literature, and there was a lack of evaluation of the long-term efficacy. (6) Because of the particularity of psychotherapy, there are obvious differences in the treatment methods between the two groups, which cannot be completely double-blind. (7) All clinical observation trials were completed in China. Due to cultural background and ethnic differences, it is uncertain whether the research results are consistent with other races or countries. The above factors may bias the experimental results and ultimately affect the experimental results.

TD is a neuropsychiatric disorder that occurs in adolescence [26], which not only affects the quality of life of children but also damages their psychology. At present, the treatment scheme for TD mainly adopts western medicine to control the clinical symptoms of TiC [27–29]. Among the 14 studies included in this study, the control group included antipsychotics such as haloperidol and tiapride, central *α*-receptor agonists such as clonidine, and antiepileptic drugs such as topiramate. It is used in the treatment of children's TD, but the side effects are obvious. With the research on the biological social psychological treatment mode of children's TD treatment, most scholars believe that children's tic disorder is related to multiple factors such as genetic factors, unbalanced level of behavioral, and psychological development [30]. Psychological intervention for young children can improve children's self-regulation ability, eliminate negative psychology, and relieve tic symptoms. Therefore, psychotherapy has a good application prospect as an adjuvant treatment for tic in children.

The results of this study show that psychotherapy combined with drugs can improve the effective rate of tic disorder and improve the clinical symptoms of TD children, but the evidence is limited and the observation of adverse reactions is insufficient. Due to the low methodological quality, the authors cautiously believe that clinical decisions should be made based on the comprehensive situation of individual children and guided by the recommendations of experts and professional organizations in the field. At the same time, it is also necessary to carry out multicenter, large sample, and multiethnic RCT research on TD; adopt strict inclusion criteria, exclusion criteria, diagnostic criteria, efficacy criteria, and treatment schemes; clarify the random method, blind method, and fully hidden distribution method; and verify the research results. It is expected that more high-quality clinical studies designed based on modern evidence-based medicine system and epidemiological methods can comprehensively, systematically, and objectively evaluate the clinical efficacy of psychotherapy combined with western medicine in the treatment of TD, and provide a reliable basis for the new methods of clinical treatment of TD.

## Figures and Tables

**Figure 1:** Document screening flow chart.

**Figure 2:** Meta-analysis forest chart of total effective rate in two groups.

**Figure 3:** Meta-analysis forest diagram of YGTSS score after treatment in two groups.

**Figure 4:** Funnel diagram of efficiency index.

**Table 1:** Methodological evaluation and bias risk assessment of included literature.

Paper source	Methods of randomization	Allocation concealment	Blind method	Lost visit/exit	Other bias	Jadad (score)
Wu et al. [12] 2021	Random digital table method	Not described	Not described	Not described	Not clear	2
Yang [13] 2020	Random digital table method	Not described	Not described	Not described	Not clear	2
Zhang et al. [14] 2020	Random digital table method	Not described	Not described	Not described	Not clear	2
Chen [15] 2020	Computer random method	Not described	Not described	Not described	Not clear	2
Yu et al. [16] 2019	Random words	Not described	Not described	Not described	Not clear	1
Dai et al. [17] 2018	Random words	Not described	Not described	Not described	Not clear	1
Li [18] 2017	Random digital table method	Not described	Not described	Not described	Not clear	2
Shi and Wang [19] 2017	Random words	Not described	Not described	Described	Not clear	2
Peng et al. [20] 2016	Random words	Not described	Not described	Not described	Not clear	1
Zhao [21] 2014	Random words	Not described	Not described	Not described	Not clear	1
Guo et al. [22] 2013	Random words	Not described	Not described	Not described	Not clear	1
Chen and Chen [23] 2017	Random digital table method	Not described	Not described	Not described	Not clear	2
Fang et al. [24] 2016	Random words	Not described	Not described	Not described	Not clear	1
Zheng et al. [25] 2014	Random digital table method	Not described	Not described	Not described	Not clear	2

Notes: random words: only random words are proposed in the text, but no specific random methods are proposed.

**Table 2:** General information of literature.

Paper source	Sample number				Age		Intervention study	
	*T*	*n* F/M	*C*	*n* F/M	*T*	*C*	*T*	*C*
Wu 2021	40	24/16	40	26/14	8.20 ± 2.25	8.76 ± 2.10	A + B	B
Yang 2020	43	29/1	43	28/15	8.72 ± 2.43	8.87 ± 2.17	A + C	C
Zhang 2020	40	31/9	40	30/10	8.78 ± 1.06	8.87 ± 1.21	A + D	D
Chen 2020	150	89/61	150	85/65	7.6 ± 2.5	7.7 ± 2.7	A + H	H
Yu 2019	50	26/24	50	25/25	5.0 ± 1.5	5.1 ± 1.3	A + C	C
Dai 2018	25	10/15	25	12/13	10.08 ± 1.76	9.67 ± 1.44	A + G	G
Li 2017	60	41/19	60	36/24	7.5	7.6	A + G	G
Shi 2017	10	8/2	21	15/6	9.30 ± 0.70	10.33 ± 1.57	A + B	B
Peng 2016	46	34/12	41	31/10	9.61 ± 2.54	9.74 ± 2.66	A + E	E
Zhao 2014	30	18/12	30	19/11	11.6 ± 3.2	10.6 ± 2.1	A + E	E
Guo 2013	50	32/18	50	33/17	10.3 ± 2.4	10.1 ± 2.9	A + G	G
Chen 2017	38	26/12	47	33/14			A + F	F
Fang 2016	25	20/5	25	18/7	8.47 ± 2.43	7.70 ± 1.77	A + D	D
Zheng 2014	36	27/9	36	26/10			A + C	C

Notes: T: treatment group; C: control group; A: psychobehavioral therapy; B: italprid; C: topiramate; D: haloperidol; E: tiapride hydrchloride; F: clonidine; G: aripiprazole; H: methylphenidate hydrochloride.

## Data Availability

The data underlying the results presented in the study are available within the manuscript.
